# Text Mining-Based Drug Discovery in Osteoarthritis

**DOI:** 10.1155/2021/6674744

**Published:** 2021-04-14

**Authors:** Rong-Guo Yu, Jia-Yu Zhang, Zhen-Tao Liu, You-Guang Zhuo, Hai-Yang Wang, Jie Ye, Nannan Liu, Yi-Yuan Zhang

**Affiliations:** ^1^Department of Orthopedics, Fuzhou Second Hospital Affiliated to Xiamen University, Fuzhou 350007, Fujian, China; ^2^School of Clinical Medicine, Yunnan University of Traditional Chinese Medicine, Kunming 650032, Yunnan, China; ^3^College of Integrated Chinese and Western Medicine, Fujian Univerisity of Traditional Chinese Medicine, Fuzhou 350122, Fujian, China

## Abstract

**Background:**

Osteoarthritis (OA) is a chronic and degenerative joint disease, which causes stiffness, pain, and decreased function. At the early stage of OA, nonsteroidal anti-inflammatory drugs (NSAIDs) are considered the first-line treatment. However, the efficacy and utility of available drug therapies are limited. We aim to use bioinformatics to identify potential genes and drugs associated with OA.

**Methods:**

The genes related to OA and NSAIDs therapy were determined by text mining. Then, the common genes were performed for GO, KEGG pathway analysis, and protein-protein interaction (PPI) network analysis. Using the MCODE plugin-obtained hub genes, the expression levels of hub genes were verified using quantitative real-time polymerase chain reaction (qRT-PCR). The confirmed genes were queried in the Drug Gene Interaction Database to determine potential genes and drugs.

**Results:**

The qRT-PCR result showed that the expression level of 15 genes was significantly increased in OA samples. Finally, eight potential genes were targetable to a total of 53 drugs, twenty-one of which have been employed to treat OA and 32 drugs have not yet been used in OA.

**Conclusions:**

The 15 genes (including PTGS2, NLRP3, MMP9, IL1RN, CCL2, TNF, IL10, CD40, IL6, NGF, TP53, RELA, BCL2L1, VEGFA, and NOTCH1) and 32 drugs, which have not been used in OA but approved by the FDA for other diseases, could be potential genes and drugs, respectively, to improve OA treatment. Additionally, those methods provided tremendous opportunities to facilitate drug repositioning efforts and study novel target pharmacology in the pharmaceutical industry.

## 1. Introduction

OA is a chronic and degenerative joint disease that occurs commonly in the elderly, and the main concomitant symptoms were cartilage loss, subchondral bone sclerosis, synovitis, and pain [1, 2]. The incidence of OA is increasing around the world due to the aging population and the growing number of obese individuals [3]. According to the statistics, the incidence of OA can reach nearly half of people over age 65 and 80% of those over age 80 [4].

There are different management methods between the end stage and early stage for OA. Traditionally, the treatments of end-stage OA for improving function and relieving pain have been joint operation [5], which may have long-term problems and potential complications, such as pain, infection, hemorrhage, and arthrofibrosis [6]. Therefore, early treatment is particularly important. Comprehensive clinical practice guidelines by the American Academy of Orthopaedic Surgeons held that NSAIDs were appropriate for all nonsurgical treatment OA patients [7]. Using the drug of NSAIDs in the treatment of OA has also been approved by the American College of Rheumatology and other academic institutions [8].

NSAIDs include traditional NSAIDs and new COX-2 inhibitors; the former blocks COX-1 and COX-2 but the new one only blocks the COX-2 enzyme. The formation of prostaglandinH2 (PGH2) by the metabolic process of the COX enzyme is metabolized by prostaglandin E (PGE) synthase into PGE2, which is one of the significant inflammation mediator [9]. COX-1, found in most tissues, is encoded by prostaglandin-endoperoxide synthase 1 (PTGS1) and COX-2, induced by various cytokines and growth factors, is encoded by prostaglandin-endoperoxide synthase 2 (PTGS2) [10]. COX-1 NSAIDs are associated with more gastrointestinal side effects than COX-2 [11], but likely have a lower rate of cardiovascular events [12]. In clinical practice, diclofenac, one kind of NSAIDs (inhibiting COX-1 and COX-2), is used as the most effective for OA treatment [4] and increases the rating of the risk of a cardiovascular event by fourfold, stroke by threefold, and all-cause death by twofold [13]. A long-term use of Ibuprofen (also inhibiting COX-1 and COX-2) shows more than three times the incidence of stroke complications compared with placebo [13]. Although there are significant limitations and health risks, approximately 65% of patients are provided oral NSAIDs to control OA [14]. After consuming NSAIDs chronically, most patients still report persistent pain and disability, and more than half will receive a prescription to stop using within one year [15]. Given all that, the securities of NSAIDs are problems that have to be paid attention to. It is still limited to research into drug therapy, and we need further studies to fill the vacancies in the development of novel therapeutic drugs.

Discovering new drug therapies is typically a 7–12 years process. With the development of computer technology and biotechnology, the article type of text mining for new drugs is becoming more common worldwide. Besides, abundant clinical trials and investment of billions of dollars are recommended but what we got are unpredictable returns on investment [16]. However, it is a less costly and possibly quicker alternative that the existing drugs are beyond their original intent to treat a novel situation [17]. Text mining of biomedical literature is a well-established approach in revealing new associations between pathologies and genes [18]. In recent years, approximately 30% of the newly Food and Drug Administration (FDA) approved vaccines and drugs are repurposing discoveries in the US [19]. As a classic example, sildenafil (Viagra), originally targeted towards angina, is used in the treatment of erectile dysfunction in men in 1998 [20].

In this study, we use bioinformatics methods to investigate novel drugs for OA. Firstly, we made a preliminary list of candidate genes for further analysis by mining text. Next, we analyzed the characteristics of genes selected by way of GO and KEGG enrichment analysis. Then, we acquired the association between those genes by PPI analysis and generated focused target genes set by the MCODE plugin. Finally, candidate key drugs were discovered from the final genes set through the drug-gene interaction analysis.

## 2. Materials and Methods

### 2.1. Text Mining

The web-based service pubmed2ensembl (http://pubmed2ensembl.ls.manchester.ac.uk/) was used to perform text mining. The link is a publicly available resource database, including biological articles from MEDLINE life science journals and online books, and linking over 2,000,000 literature to nearly 150,000 genes from 50 species [21]. All gene names, related to the search concepts found in the available literature, are extracted from pubmed2ensembl when a query is performed [21]. In this study, we performed queries using the search terms (*Osteoarthritis and NSAIDs*) for producing two gene lists. Common unique genes between the two lists were then used to proceed to the next steps.

### 2.2. Biological Process and Pathway Analysis

We used the FUNRICH (http://www.funrich.org) for a GO enrichment analysis, including biological process (BP), cellular component (CC), molecular function (MF). FUNRICH is a stand-alone software tool whose one kind of function is for the functional enrichment of genes and proteins. The KEGG pathway analysis was performed with annotations (chemokine activity, catalytic activity, transcription factor activity, receptor activity, growth factor, receptor binding, and cytokine activity) from the DAVID (Database for Annotation, Visualization, and Integrated Discovery), which contained all the gene terms we mined. DAVID (https://david.ncifcrf.gov/summary.jsp) is a web-based tool, providing functional annotation tools for the researcher to understand biological meaning among a large list of genes.

### 2.3. Protein Interaction Network

We used the STRING database (http://string-db.org) for acquiring a key estimation of protein-protein functional associations. The study reported that this database could comprehensively integrate the PPI of selected genes. Then, we used the MCODE (molecular complex detection) plugin of Cytoscape (version 3.7.1) to seek a gene list of the tightest interaction network among all common genes. The parameters of MCODE were used: node score cutoff ≥0.05, degree cutoff ≥2, maximum depth = 100, and k-score ≥2 [22].

### 2.4. Quantitative Real-Time- (qRT-) PCR Array Validation

To validate the findings of bioinformatics analysis, synovial tissues from patients were harvested for qRT-PCR validation between the OA group (*n* = 8) and the control group (*n* = 8). The use of verbal consent was approved by Fuzhou Second Hospital affiliated to Xiamen University, and oral consent was obtained by each subject. Total RNA from the lesion of synovial tissue was extracted using TRIzol reagent (TAKARA, Dalian, China). RNA samples from total RNA were reverse-transcribed to cDNA using the Revert Aid First Strand cDNA Synthesis Kit (TaKaRa, Japan) according to the manufacturer's instructions. The conditions were set as follows: 95°C for 30 sec for denaturation, cycling stage 95 °C/10 s, and 60 °C/0.5 minutes (40 cycles). GAPDH was then handled as an internal reference. Relative mRNA expression was calculated using the 2-ΔΔCt method. *P* values < 0.05 indicated a significant difference. The sequences of primers are presented in Table 1.

### 2.5. Drug-Gene Interactions

The web-based Drug-Gene Interaction Database (DGIdb) (version 3.0, http://www.dgidb.org) was used to search drug-gene interactions of the confirmed genes, which might cause associations with small organic compounds or drugs. The DGIdb aggregates drug-gene interaction data from 27 kinds of sources, including PharmGKB, DrugBank, NCBI Entrez, ChEMBL, PubChem, Ensembl, and other authoritative databases. It organized the results of the search so that drug-gene interaction was available to match with relevant gene entry by its source link [23].

## 3. Results

### 3.1. Text Mining and Biological Process

Based on the strategy of data investigation described in Figure 1, from text-mining searches by pubmed2ensembl, we determined 550 unique genes (Figure 2), related to both OA and NSAIDs (we do not rule it out that some of them may have more than one name). All gene names are shown in Appendix S1. In the process of GO biological annotations, we are based on the characteristics of the results from data analysis in FUNRICH. The cellular-components annotations revealed that most of the genes are expressed in the Cytoplasm (51.1%), plasma membrane (46.6%), and extracellular (32.5%), and other details are seen in Figure 3. The GO enrichment analysis of molecular functions (transmembrane receptor protein tyrosine kinase activity, G-protein coupled receptor activity, receptor activity, growth factor activity, receptor binding, chemokine activity, protein serine/threonine kinase activity, and cytokine activity) demonstrated that 7.5% of the identified genes had G-protein coupled receptor activity (Figure 4). Biological process annotations showed cell communication (35.1%) and signal transduction (39%) were the most highly enriched terms (Figure 5).

### 3.2. Pathway Analysis

For the procedure of KEGG pathways enrichment analysis, more enriched genes and relatively low *P* values showed that the pathways are particularly relevant to OA and NSAIDs. The four most enriched biological KEGG pathway were (1) pathways in cancer (5.49E-36); (2) TNF signaling pathway (2.45E-26); and (3) proteoglycans in cancer (1.86E-21), PI3K-Akt signaling pathway (6.99E-21), containing 101, 46, 56, and 74 genes related to pathways enrichment analysis, respectively, and other highly enriched pathways including FoxO signaling pathway, HIF-1 signaling pathway, MAPK signaling pathway, prolactin signaling pathway, osteoclast differentiation, apoptosis, chemokine signaling pathway, and Toll-like receptor signaling pathway. To more intuitively present the details, we conducted mapping with R statistical software (version 3.6.1) (Figure 6).

### 3.3. Protein-Protein Interaction

The protein-protein interaction analysis was performed using STRING and we set the following parameters: (1) minimum required interaction score: medium confidence (0.400) and (2) display simplifications: hide disconnected nodes in the network. Network Stats showed the results: the number of nodes: 452; the number of edges: 11095; average node degree: 49.1; local clustering coefficient: 0.529; expected number of edges: 4532; and PPI enrichment *P* value: <1.0e-16 (Figure 7). Then, the data format “.tsv” was imported from the STRING EXPORTs channel to the MCODE plugin of Cytoscape and the following parameters were set: node score cutoff: 0. 05; K- -core: 2; max. depth: 100. Based on these criteria, we selected 22 central genes which formed the tightest module network, including PTGS2, NLRP3, MMP13, MMP9, IL1RN, CCL2, CXCL8, TNFRSF1B, TNF, CASP3, IL10, CD40, MAPK8, STAT3, IL6, NGF, TP53, RELA, BCL2L1, VEGFA, NOTCH1, and HMGB1 (Figure 8). We used DAVID to perform KEGG pathways enrichment analysis of central genes and picked the top 10 most enriched biological KEGG pathways to list out in Table 2 (Table 2). From Table 2, it is not difficult to find that all of those genes are involved in the enriched pathways.

### 3.4. qRT-PCR Validation of the Hub Genes

A qRT-PCR approach was used to detect the expression levels of 22 potential genes. The verification result showed that the expression levels of PTGS2, NLRP3, MMP9, IL1RN, CCL2, TNF, IL10, CD40, IL6, NGF, TP53, RELA, BCL2L1, VEGFA, and NOTCH1 were significantly increased in osteoarthritis samples (*P* < 0.05) (Figure 9), which confirmed the analytical results of bioinformatics were reliable in this study.

### 3.5. Drug-Gene Interactions

The final confirmed genes were used to conduct drug-gene interaction analysis, and a list of 53 drugs was regarded as potentially meeting possible drug therapy for OA (Table 3). Potential gene targets of the drugs in this list are PTGS2 (35 drugs), TNF (7 drugs), VEGFA (5 drugs), MMP9 (2 drugs), and CCL2, IL1RN, IL6, and NGF (1 drug each). 21 of 53 drugs have been employed to treat OA and 32 drugs (including 16 drugs target COX-2) have not yet been used in OA. The interrelation of the 32 drugs with genes and pathways is shown in Figure 10.

## 4. Discussion

As the obesity rate and ages of the world population increase, the morbidity of OA is increasing especially in older adults. OA is one of the most common conditions causing decreased function, joint pain, and stiffness. To relieve symptoms by the improvement of joint function and reduction of pain, the classical treatment of OA is still using NSAIDs [24]. However, the long-term use of NSAIDs sometimes may cause headaches, gastrointestinal disturbances, and cardiovascular side effects. To address this question, we utilized bioinformatics tools to identify existing potential NSAIDs for OA treatment. Consequently, we identified eight targeting potential genes and 53 drugs associated with OA (Table 3).

The exact mechanism of OA pathogenesis remains to be elucidated, but the inflammation and cartilage degradation is the main pathological feature of OA [25]. The mechanism at a molecular level of inflammation and cartilage destruction involves multiple factors, such as matrix metalloproteinases (MMPs), COX-2, and ADAMTS (a disintegrin and metalloproteinases with thrombospondin motifs), in articular chondrocytes [26]. Mechanical stress, proinflammatory cytokines (including tumor necrosis factor-*α* (TNF-*α*), and interleukin-6 (IL-6), IL-17, IL-1*β*) can promote COX-2 and ADAMTS expression and accelerate the destruction of cartilage and OA development. PGE2 that is associated with the activity of TNF-*α* and IL-1*β* can lead to a large reduction in proteoglycan content in cartilage tissue [27]. The MMPs (especially 1 and 13) play major roles in cartilage matrix degradation and result in focal lesions in the articular surface [28]. Several studies reported increased expression of MMP-13 in OA. This difference may be caused as follows: PCR stochasticity, primer biases, multiple species in individual samples, and pooling of samples exerts too many uncertainties that could bias the results. Additionally, the sample size was insufficient. Proinflammatory cytokines can increase in nitric oxide (NO) and PGE2 synthesis and release [29]. Previous studies have shown that the anti-inflammatory effects of NSAIDs mainly depend on the function of inhibiting COX, reducing the generation of prostaglandins, which are the major mediator of pain and inflammatory response [30, 31].

In our results, the PTGS2 gene responsible for encoding COX-2 is corresponding to the most diverse class of drugs. Among them, 20 drugs are not applied for the treatment of OA but have been approved by the FDA to treat other diseases and obtained excellent outcomes. The mesalamine (5-ASA) compounds are commonly well tolerated and rare complications [32]. In the European [33] and the United States [34] guidelines, 5-ASA was recommended as a frontline agent for treating patients with mildly to moderately active ulcerative colitis. From the molecular structures' point of view, the intensity of halogenation is positively correlated with drug therapy strength. It is considered that such a difference may also allow bromfenac (containing a bromine atom) wider ocular distribution [35]. Bromfenac is better than both dexamethasone and fluorometholone in preventing cystoid macular edema [36]. Although the molecular mechanism of sulfasalazine remained ambiguous, the drug is known to play a role that is immunomodulatory and anti-inflammatory [37]. It has also been the widely used treatment of other diseases, such as and ulcerative colitis, Crohn's disease, and ankylosing spondylitis [34, 38, 39].

The platelet-derived growth factor superfamily secreted vascular endothelial growth factor A (VEGFA), a glycoprotein that mediates glomerular endothelial cell biological functions [40]. Glomerular visceral epithelial cells, known as podocytes, secrete VEGFA, a glycoprotein that mediates glomerular endothelial cell biological functions [40]. In the early stages of diabetes, podocytes increasing the expression of Vegfa can lead to both insulin deficiency and resistance in rodents [41]. Furthermore, Vegfa is also irreplaceable to induce the formation of cartilage. A significant positive correlation between the overexpression of Vegfa in osteochondrogenic cells and bone mass is also observed [42]. At the early stage of bone development, Vegfa was regarded as a regulator of both osteoblast differentiation and perichondrial vascularity [43].

There were also some limitations to the study. Firstly, the databases we used may be limited to get accurate information on genes concerning function or role. With the databases becoming more comprehensive, the results of the analysis will be more accurate. Although we have validated results in multiple biological databases, further molecular biological experiments of the large sample are indispensable to confirm the reliability of the results. We cannot ensure that a given gene is known to all relations of existing drugs and drug-gene interactions. Therefore, it is possible that we missed or ignored the drugs which could potentially be useful.

## 5. Conclusion

In conclusion, we have presented a way to investigate the potential candidate drugs which target the genes/pathways relevant to OA. With the databases and analytical tools evolved and improved, such a method may be used routinely to explore more diseases and to facilitate drug repositioning efforts in the pharmaceutical industry. From the present analysis, we identified a total of 53 potential drugs, of which 32 drugs targeted other OA-relevant pathways but have not yet been used in OA, which could give us a clue to novel therapeutic targets as potential treatments for OA. However, further direct evidence by molecular biological experiments is necessary to make clear their association with OA.

## Figures and Tables

**Figure 1:** Overall data mining strategy. Text mining was used to identify genes associated with the concepts of OA and NSAID using pubmed2ensemble. Extracted genes were then analyzed for their function and gene ontology using Funrich. Further enrichment was obtained by molecular network analysis using STRING and Cytoscape. The final enriched gene list was then used to determine interactions with known drugs using the Drug Gene Interaction Database.

**Figure 2:** A Venn diagram showing the overlapping genes between OA and NSAIDs.

**Figure 3:** The cellular-component annotations of those gene sets.

**Figure 4:** The molecular functions annotations of those gene sets.

**Figure 5:** The biological process of those gene sets.

**Figure 6:** The enriched biological KEGG pathway.

**Figure 7:** Protein-protein interaction (PPI) network of common genes.

**Figure 8:** The tightest module from the PPI network.

**Figure 9:** RT-PCR validation of the hub gene between OA and normal controls.

**Figure 10:** The interrelation of 32 drugs with genes and pathways.

**Table 1:** Lists of primer sequences used for quantitative real-time PCR.

Genes	Sequences	
	Forward	Reverse
PTGS2	CCGAGGTGTATGTATGAGTG	GGGAGGGAGAAATTAATGGG
NLRP3	CACAGTCTAGTTGGGAAGAC	GAGACCATGTCTTCCATCAC
MMP13	CTTCCTCTTCTTGAGCTGG	GCAAGATACTCTACCTCTGC
MMP9	ATGTCTAAGGAGGGGAGATC	CTCAAACTCCTGAGCTTCAG
IL1RN	CTGGTATGTTCCTGTGGAAG	GGATAGGAGGCAGGACTAAT
CCL2	GTAATCAAAGAGAGGGTGGG	CTCATTACCTCTGCAGAGTC
CXCL8	CAAGCTTCTAGGACAAGAGC	CTTACCTTCACACAGAGCTG
TNFRSF1B	GGGCTGTCAGACTAGAATTG	CAGAGTATATGGCATGACCC
TNF	GAAGACACTCAGGGAAAGAG	TGATTAGAGAGAGGTCCCTG
CASP3	CAGGCAGAGGGATCTTTATG	CACTAGGTATGAAGGTCAGC
IL10	GCTTCTTAATCCCTGGGATC	CTCAGTCCTGGTCTTCTTTC
CD40	CCAAAGGTCTCATAGCTAGC	GTTCTCACTCCCCATAGTTC
MAPK8	GAGGTCAGATGCTCTAAGTG	CTATATTCCAGGCTAGGTGG
STAT3	CTGAAAGACTTCATGGGAGG	CCTCACTTCCCAAGTTAGAC
IL6	CGTCCGTAGTTTCCTTCTAG	AGGGGGAGAATACTACTCAC
NGF	CTCTTGTTGAAGGGGGATAG	CTCTGAGGTGCTCCTATACT
TP53	GATGAGTCCTCTCTGAGTCA	GTCCTAACATCCCCATCATC
RELA	CTATGAAGTAGCCGCTACAG	GAAGTGATTAGGGACCCATC
BCL2L1	TAGACCCAGACCTTCGTAAG	GAAGGGAGAGAAAGAGCTTC
VEGFA	CAGTGCTAGGAGGAATTTCC	CAGTGATCATCCTTTCCCTG
NOTCH1	GGCGAGAATTATCTGTCCTC	GGATCAATTACTCAAGCCCC
HMGB1	CAGGAGATCAGCAGAGATTG	CTGGGACCAGGATATGTAGA

**Table 2:** Summary of KEGG pathways gene set enrichment analysis.

Pathways	Genes in query set	Total genes in genome	Percentage (%)	*P* value	Genes
TNF signaling pathway	9	108	0.267857	1.73E-10	CASP3, TNFRSF1B, IL6, TNF, CCL2, PTGS2, RELA, MMP9, MAPK8
NOD-like receptor signaling pathway	7	166	0.208333	5.53E-09	IL6, TNF, CCL2, RELA, CXCL8, MAPK8, NLRP3
Pathways in cancer	11	515	0.327381	1.92E-08	CASP3, IL6, PTGS2, RELA, MMP9, VEGFA, TP53, CXCL8, MAPK8, BCL2L1, STAT3
Apoptosis	6	135	0.178571	5.33E-07	CASP3, TNF, RELA, TP53, BCL2L1, NGF
NF-kappa B signaling pathway	6	93	0.178571	2.91E-06	TNF, PTGS2, RELA, CXCL8, BCL2L1, CD40
Toll-like receptor signaling pathway	6	102	0.178571	7.74E-06	IL6, TNF, RELA, CXCL8, MAPK8, CD40
Amyotrophic lateral sclerosis (ALS)	5	50	0.14881	8.84E-06	CASP3, TNFRSF1B, TNF, TP53, BCL2L1
Inflammatory bowel disease (IBD)	5	62	0.14881	2.38E-05	IL6, TNF, RELA, IL10, STAT3
Cytokine-cytokine receptor interaction	7	263	0.208333	3.37E-05	TNFRSF1B, IL6, TNF, CCL2, CXCL8, CD40, IL10
Adipocytokine signaling pathway	5	69	0.14881	3.40E-05	TNFRSF1B, TNF, RELA, MAPK8, STAT3

To make sure that only the most enriched annotations were selected, a *P* value cutoff (*P*=1.00*E* − 05) was set. Among the most significantly enriched pathway annotations above the cutoff, those most relevant to OA pathology based on the available literature and research were selected. A total of 10 pathways were picked out from the analysis of enriched pathway annotations.

**Table 3:** Candidate drugs targeting genes with OA.

Number	Drug	Description	Gene	Drug-gene interaction	Score	Approved by FDA	Approved use in OA	Clinical trial phase in O A	Reference (PubMed ID)
1	Celecoxib	COX-2	PTGS2	Inhibitor	12	Yes	Yes	4	12093311|12086292
2	Etodolac	Mainly COX-2	PTGS2	Inhibitor	11	Yes	Yes	2	12824918|11009046
3	Oxaprozin	Mainly COX-1	PTGS2	Inhibitor	10	Yes	Yes	2	19338579|9831331
4	Meloxicam	COX-2	PTGS2	Inhibitor	11	Yes	Yes	4	10567199|10220944
5	Icosapent	Eicosanoids	PTGS2	Inhibitor	7	Yes	No	Not available	12573452|16190133
6	Aminosalicylic acid	Antimycobacterial agent	PTGS2	Inhibitor	6	Yes	No	Not available	16855178|12463455
7	Mesalamine	Anti-inflammatory agent	PTGS2	Inhibitor	9	Yes	No	Not available	16855178|12463455
8	Indomethacin	Mainly COX-1	PTGS2	Inhibitor	8	Yes	Yes	4	15668944|15730717
9	Nabumetone	COX-2	PTGS2	Inhibitor	11	Yes	Yes	4	11304699|12047490
10	Tenoxicam	PTG synthetase inhibitor	PTGS2	Inhibitor	10	Yes	Yes	2	11563332|16245223
11	Lenalidomide	Immunomodulatory drug	PTGS2	Modulator	3	Yes	No	Not available	15598423|12720152
12	Rofecoxib	COX-2	PTGS2	Inhibitor	15	Yes	Yes	3	10580458|11398914
13	Piroxicam	COX-1	PTGS2	Inhibitor	10	Yes	Yes	2	11952155|11785774
14	Sulindac	PTG synthetase inhibitor	PTGS2	Inhibitor	9	Yes	Yes	2	11118042|10372826
15	Mefenamic acid	PTG synthetase inhibitor	PTGS2	Inhibitor	11	Yes	Yes	2	10393680|15792781
16	Naproxen	PTG synthetase inhibitor	PTGS2	Inhibitor	11	Yes	Yes	4	17604186|17612049
17	Sulfasalazine	PTG synthetase inhibitor	PTGS2	Inhibitor	7	Yes	No	Not available	16855178|12463455
18	Phenylbutazone	PTG synthetase inhibitor	PTGS2	Inhibitor	9	Yes	No	Not available	15939622|15489888
19	Diflunisal	PTG synthetase inhibitor	PTGS2	Inhibitor	11	Yes	Yes	Not available	11315375|8737748
20	Suprofen	PTG synthetase inhibitor	PTGS2	Inhibitor	7	Yes	No	Not available	11885959|17139284
21	Salicylic acid	PTG synthetase inhibitor	PTGS2	Inhibitor	10	Yes	Yes	Not available	15035793|15348270
22	Aspirin	Mainly COX-1	PTGS2	Inhibitor	12	Yes	Yes	Not available	17522398|17181859
23	Bromfenac	PTG synthetase inhibitor	PTGS2	Inhibitor	6	Yes	No	Not available	16982289|16846546
24	Ketoprofen	COX-2	PTGS2	Inhibitor	11	Yes	Yes	3	14513718|11729362
25	Balsalazide disodium	PTG synthetase inhibitor	PTGS2	Inhibitor	7	Yes	No	Not available	17981262|12950415
26	Lumiracoxib	COX-2	PTGS2	Inhibitor	10	Yes	Yes	3	14965322|15017615
27	Salsalate	PTG synthetase inhibitor	PTGS2	Inhibitor	7	Yes	Yes	Not available	9711054|10452868
28	Ginseng, Asian	Adaptogen	PTGS2	Inhibitor	4	Yes	No	Not available	17436372|15753395
29	Antrafenine	Cyclooxygenase inhibitor	PTGS2	Inhibitor	7	Yes	No	Not available	17604186|17612049
30	Antipyrine	Cyclooxygenase inhibitor	PTGS2	Inhibitor	2	Yes	No	Not available	11695253
31	Tiaprofenic acid	PTG synthetase inhibitor	PTGS2	Inhibitor	8	Yes	Yes	Not available	2277128|11752352
32	Etoricoxib	COX-2	PTGS2	Inhibitor	12	Yes	Yes	4	17573128|17164136
33	Resveratrol	Polyphenolic phytoalexin	PTGS2	Inhibitor	2	Yes	No	3	11752352
34	Nepafenac	COX-1 and COX-2	PTGS2	Inhibitor	5	Yes	No	Not available	10850857
35	Parecoxib	COX-2	PTGS2	Inhibitor	3	Yes	No	Not available	10794682
36	Captopril	Inhibitor of ACE	MMP9	Inhibitor	5	Yes	No	Not available	12381651|19057128
37	Glucosamine	Precursor of lipids	MMP9	Antagonist	6	Yes	Yes	4	12405690|16616490
38	Rilonacept	Interleukin 1 inhibitor	IL1RN	Binder	3	Yes	No	Not available	23319019|12815153
39	Danazol	Gonadotropin inhibitor	CCL2	Inhibitor	3	Yes	No	Not available	11056242|11216879
40	Etanercept	Fusion protein	TNF	Antibody	12	Yes	No	Not available	10375846|10405518
41	Adalimumab	Monoclonal antibody	TNF	Antibody	12	Yes	No	Not available	12044041|15022409
42	Infliximab	TNF-*α* blocker	TNF	Inhibitor	17	Yes	No	Not available	16456024|16052578
43	Inamrinone	PDE3 inhibitor	TNF	Inhibitor	6	Yes	No	Not available	11805217|1611705
44	Golimumab	Monoclonal antibody	TNF	Antibody	6	Yes	No	Not available	21079302
45	Certolizumab pegol	TNF-*α* inhibitor	TNF	Neutralizer	6	Yes	No	Not available	23620660
46	Pomalidomide	COX-2	TNF	Inhibitor	2	Yes	No	Not available	22917017
47	Siltuximab	Monoclonal antibody	IL6	Antagonist	4	Yes	No	Not available	8823310
48	Clenbuterol	Beta(2) agonist	NGF	Stimulator	6	Yes	No	Not available	10525174|10403429
49	Aflibercept	Recombinant fusion protein	VEGFA	Inhibitor	7	Yes	No	Not available	22813448
50	Carvedilol	Beta adrenoceptor blocker	VEGFA	Other	5	Yes	No	Not available	15071347|15942707
51	Dalteparin sodium	Anticoagulant	VEGFA	Inhibitor	4	Yes	No	Not available	17692905|21091776
52	Ranibizumab	VEGFA antagonist	VEGFA	Inhibitor	14	Yes	No	Not available	18046235|18054637
53	Bevacizumab	VEG inhibitor	VEGFA	Inhibitor	10	Yes	No	Not available	15705858|11752352

Fifty-three drugs which met the criteria of targeting one of the candidate genes by an appropriate interaction were collected in the final list. Whether the drug has been approved by the FDA and whether it has been approved for OA are documented in the table. ACE: angiotensin-converting enzyme; TNF: tumor necrosis factor; PDE: phosphodiesterase; PTG: prostaglandin; VEGF: vascular endothelial growth factor.

## Data Availability

The data used to support the findings of this study are included within the supplementary information file.

## Abbreviations

OA: Osteoarthritis
NSAIDs: Nonsteroidal anti-inflammatory drugs
GO: Gene ontology
KEGG: Kyoto Encyclopedia of Genes and Genomes
PPI: Protein-protein interaction
COX: Cyclooxygenase
PGH2: Prostaglandin H2
PGE: Prostaglandin E
PTGS1: Prostaglandin-endoperoxide synthase
PTGS2: Prostaglandin-endoperoxide synthase
FDA: Food and Drug Administration
BP: Biological process
CC: Cellular component
MF: Molecular function
DGIdb: Drug-Gene Interaction Database
MMPs: Matrix metalloproteinases
TNF-*α*: Tumor necrosis factor-*α*
IL: Interleukin
NO: Nitric oxide
VEGFA: Vascular endothelial growth factor A.

## Supplementary Materials

Supplementary Materials All gene names are shown in Appendix S1.
